RETRACTED

# Effectiveness of Artificial Intelligence (AI) in Improving Pupils' Deep Learning in Primary School Mathematics Teaching in Fujian Province

**DOI:** 10.1155/2022/1362996

**Published:** 2022-09-23

**Authors:** Yaping Qiu, Junjie Pan, Nor Asniza Ishak

**Affiliations:** ^1^Chengyi University College, Jimei University, Xiamen, Fujian 361000, China; ^2^School of Educational Studies, University Sains Malaysia, 11800 USM, Penang, Malaysia

## Abstract

Several primary school students in Fujian Province have perceived studying mathematics as challenging. To deal with this issue, computer technology advancements, specifically artificial intelligence (AI), present an opportunity to evaluate individual students' learning challenges and give individualized support to optimize their success in mathematics classes. It is also possible to use virtual reality (VR) to assist learners in acquiring complex mathematical and logical ideas and to lessen learners' mistakes. As a result, researchers, particularly beginners, are missing out on a complete perspective of the study of AI in teaching mathematics. That is why we are exploring the role of AI in math education by developing a “fuzzy-based tweakable convolution neural network with a long short-term memory (FT-CNN-LSTM-AM)” method. For this investigation, the students' datasets are taken and educated by mathematical teaching via the application of AI. The proposed method is utilized to predict the students' performance in mathematical education. A grey wolf optimizer is employed to boost the effectiveness of the proposed method. Furthermore, the performance of the proposed method is analyzed and compared with existing approaches to gain the highest reliability.

## 1. Introduction

Mathematics is a branch of education that uses symbolic language to represent ideas such as numbers, amounts, places, and architecture. Math education has been described as a complex and challenging undertaking to improve students' problem-solving abilities. Many prior studies have found that students typically find it extremely difficult to finish mathematical problems, particularly those that require multiple stages also to be completed. As a result, academics have attempted to create diverse learning techniques and technologies to help pupils improve their math academic achievement. They also stressed the necessity of recognizing the elements that impact students' arithmetic academic achievement, such as a lack of prior learning and individualized help for different students. Hence, advances in artificial intelligence (AI) have created a mechanism to address these issues. AI is an application of computers creating intelligent computer networks that can do tasks that need human intelligence, such as visual and communication skills, inference, and decision-making. Some past uses have shown the promise of teaching and learning, particularly for assisting the students with complicated or challenging tasks. AI may play various roles throughout education, including innovative lecturer, trainee, training device, and companion, and also an adviser for academic policymaking. In terms of an intelligent tutor role, various studies have indicated the application of AI technology to replicate instructors' intelligence and deliver individualized advice, comments, or assistance to specific students throughout the education process Hwang and Tu [1]. Under current education circumstances, fundamental mathematics instruction is based on intelligent adjustments and pays attention to promoting students' personal growth. Natural language, intelligent agents, fuzzy control, artificial neural, and automation are just a few of the topics covered by artificial intelligence. AI algorithms operate as the brains of robotics, allowing robots to act as virtual personal assistants in a computerized world.

RETRACTED

AI encourages the creation of autonomous, readily modifiable programs and addresses a few 21st-century abilities such as personality, identity, and cooperation. The increasing relevance of AI may be demonstrated in developing increasingly complex systems that can comprehend and understand speech sounds and fight at higher levels of competition Wu [2].  Figure 1 shows how artificial intelligence may improve educational results and instructors' teaching techniques. The way individuals learn and develop those new skills will be heavily influenced by AI. In one sense, “AIEd” (artificial intelligence in education) can be substantially automated and identify where a human school's support is most required. It may be helpful for instructors in determining the most successful teaching methods depending on pupils' situations and educational backgrounds. This can automate pattern recognition technique operations, make evaluations, and grade and report automatically. AI influences not just what students are learning via suggestions and how they study, where cognitive difference exists, what approaches are most successful, and how to keep kids' attention. Instructors are the “person” in these situations, and AI's function is limited to assisting teachers in making the best judgments by providing student accomplishment estimates or suggesting relevant material to children with instructor approval. In this instance, the instructors make the ultimate choice Chaudhry and Kazim [3].

Including games such as chess, checkers, Stratego, or puzzle may aid in studying mathematics. Furthermore, the students may be exposed to more subtle analyses, such as prisoner's choice. Students would have had access to a wealth of material on the Internet, so looking out the laws, tips, and methods to learn games such as chess or Go might be a fun pastime in and of itself. Studying essays or online articles about the history of the games may provide further incentive for the pupils; it would be instructive and inspiring. Their solving strategies or approximation techniques in mathematics can be used in the school. For example, mathematics games such as chess or Go may be used to develop students' logical abilities at any academic level. It may be an exciting stimulant to enhance latent possibilities in primary education, and it may help starting researchers improve their rational and logical abilities at higher levels.

RETRACTED

Tools such as graphs, which are now in use in mathematics and AI, can be used to present old and highly intriguing topics such as the halting issue and the travelling man question Malik et al. [4].

In this study, we investigate the relevance of AI in math teaching by building a fuzzy-based tweakable convolutional neural network (FT-CNN-LSTM) technique. The datasets of the students are used in this project, and they are taught mathematics using AI. To forecast students' success in math classes, the suggested approach is put to the test.

A literature review and a characterization of the issue can be found in Section 2; Section 3 outlines the suggested strategy, Section 4 details the results and discusses them, and Section 5 provides a summary and a conclusion.

## 2. Related Works

In Estevez et al. [5], they look at new techniques to teach students about the principles and functioning of two famous AI algorithms. They provide the elements of an educational usage scaffold in which learners may work just on the Clawing portion programming of the algorithms to study the behavior of an algorithm plus build knowledge of the underlying computer science of AI processes. In Mody and Bhoosreddy [6], most of these disorders have numerous odontogenic keratocysts. Several odontogenic keratocysts were found in three-year female teenagers. During the study, no further anomalies were detected. In Garg and Harita [7], the personalized health care uses perfectly alright data to identify specific deviations from the norm. Using “Virtual Twins” within a design, such emerging information healthcare systems were ethically examined.

Phenomena were digitally linked and shown on the whole of a continuous basis. Moral differences can be discerned obtained from data forms and perceptions. Virtual twins' social and ethical ramifications are investigated. Information has become increasingly important in the healthcare system. Since it provides practical ways for increasing equality and fairness, this strategy has the potential to become a societal equalizer. In Ahmed et al. and Aatiqa [8], hypersensitivity is a lengthy worldwide epidemic. Often the recommended therapies in Taiwanese medical centers are traditional Chinese or China drugs. Hay fever was the most common chronic condition treated by ambulatory conventional Chinese medicine. In Taiwan, allergic sinusitis is managed with a variety of old Chinese medicine and modern medications. In Shahabaz and Afzal [9], HDR brachytherapy has been used to reduce radiation and allow outpatient treatment and quicker testing timeframes. Adjusting the latency at each dwell site, a human generator could improve dosage dispersal even more. Because of the short treatment periods, no data validation is possible, and errors can cause harm to people, and HDR brachytherapy therapies should be performed accurately. Li [10] presented a treatment technique and equipment for residential wastewater to improve rural communities. In Salihu and Zayyanu [11] Zamfara, Nigeria, hydrophilic and organophosphate insecticides were found in soil samples collected from chosen vegetable farms. Three main uses of GC-MS are focused to assess the testing regime and outcomes.

RETRACTED

In Chassignol et al. [12], the research will utilize a bibliometric map-based assessment and scanning of the Internet. A literature review was performed to analyze AI's status and historical trends in mathematics education. The Web of Scientific (WOS) database for relevant published articles is organised in the order of items searchable by the Social Sciences Citation Index (SSCI). In Malik et al. [4], they have examined the numerous research breakthroughs conducted worldwide relating to the artificial intelligence approaches used in the educational sector to summarize and emphasize the function of AI in instruction and student assessment in this article. In Baker [13], they hypothesize on the coming days of AIED study based on three applications of education methodology: models for analytic methods, modeling as elements of instructional artifacts, and designs as grounds for instructional artifact development.

In Shin [14], this research aims to learn more about how future mathematics instructors see this need for AI and its role in future mathematics education. Consequently, potential instructors realized that using AI in mathematics instruction is a requirement of the new era, that different sorts of lessons could be applied, and that precise data and understanding could be supplied. In Ee and Huh [15], this research aims to think about the future of mathematics education in light of the changing educational model and the advancement of artificial intelligence as just a result of advances in information and communication technologies. They also looked at how artificial intelligence may be used in mathematics instruction. The paper presented and produced at the Sixth World Conference on Mathematics Education in Budapest for both the topic grouping T2 surveying presentation and the overall paper provides an overview and assessment of significant achievements in using digital information technology to develop contexts for mathematical thought [16].

RETRACTED

In Thanh and Tuan [17], the article describes a project incorporating adaptive assessments into a messenger app Chabot system to measure students' mathematical performance at Vietnamese primary schools. A quantitative research approach was carried out to examine the benefits and drawbacks of this integral model in today's teaching environment. In Deo et al. [18], the research calls for developing learning and teaching interventions and class medical checks to address concerns linked to graduation results and students ‘ learning qualities in university education. In Shen and Wu [19], the author followed with an explanation of the mathematical thinking cultivation approach. Lastly, the everyday use of mathematical thinking in artificial intelligence is thoroughly explained. It is indeed possible to further incorporate the functionality of mathematical thinking to boost unnatural intelligence growth theoretically and practically via the study of mathematical knowledge in artificial intelligence.

### 2.1. Problem Statement

Education is a complicated sort of human cognition performance, notably mathematics understanding. Long- and short-term memory, the ability to remember mathematical information, and visual-spatial awareness abilities are also factors. Those elements may have varying degrees of effect. Several factors for pupils' difficulty in mathematics learning have been discovered in previous studies. Variations in pupils' teaching mathematics are caused by cognitive, emotional, and contextual variables. School counselors looked at the link between arithmetic education and certain cognitive variables. Intellect, learning and memory, and speed of processing all have an impact on math. Inadequate teaching or learning materials, a lack of enthusiasm, and poor attitudes on the part of teachers and students are all key contributors to poor mathematics achievement. Student success has improved significantly due to parental participation and assistance from these other relatives.

RETRACTED

## 3. Proposed Methodology

A fuzzy-based tweakable convolution neural network (FT-CNN-LSTM-AM) approach is used in this article to examine the importance of AI in math education. In the design of consumer goods, where cost is a crucial factor, the fuzzy logic approach is frequently utilized. A generalized linear model (GLM) is for fundamental local picture patch and serves as the convolution filter in fundamental CNNs. When an instance of latent ideas can be linearly separated, it is effective for abstraction. Here, we describe several initiatives to improve its capacity for representation. A group of frequently connected blocks, referred to as memory blocks, make up an LSTM hidden layer. The blocks can be viewed as differentiable iterations of a computer's memory chips. Input, output, and forget gates are three multiplicative units that each comprise one or more frequently connected memory cells and continuous analogues of the operations read, write, and reset for the cells. Student data are utilized in this project, which teaches arithmetic using artificial intelligence. It is put to the test to see whether it can predict students' achievement in math courses.  Figure 2 depicts the proposed methodology.

### 3.1. Dataset

We utilize two datasets collected in 2016 from 3 separate Chinese areas. Dataset 1 was collected from 17,252 pupils in 128 elementary schools throughout “Guizhou and Jiangxi provinces.” Dataset 2 contains data on 5,900 pupils from 68 Shaanxi primary schools. The counties of “Shaanxi, Guizhou, and Jiangxi are in China's northwest, southwest, and southeast,” respectively.  Table 1 shows the dataset description Gao et al. [20].

In the provinces of Shaanxi, Guizhou, and Jiangxi, we gathered data on student age and gender. Only Shaanxi Province gathered information on student Hukou types, whereas Guizhou and Jiangxi provinces only collected information about student boarding status and family assets. Similarly, with the help of local education bureaus, a standardized mathematical examination was carefully able to ensure that test contents are acceptable for students' grade levels and in accordance with the national standards. The standardized mathematical test was then put through many rounds of pilot testing of children in grades 3 through 6 to ensure that it was relevant and had suitable time restrictions. To guarantee good distributional qualities, the psychometric properties of the tests were then confirmed using information from extensive pilot testing (no bottom or top coding, for example). As a result, we were able to guarantee that the assessments were of the greatest quality and suitable for the kids' grade levels.

RETRACTED

### 3.2. Mathematical Teaching

Teaching mathematics in primary schools examines the curricula in education institutions, emphasizing how students may connect what they learn in math to other areas of the curriculum and the world beyond the classroom. The researchers draw on the most recent global studies to show how teachers may develop a diversified repertoire of instructional tactics and proper planning, assessment, and reporting procedures. The authors explain how to build inviting classroom environments for all students while improving their mathematics ability and knowledge.

### 3.3. Application of Artificial Intelligence (AI) Using Virtual Reality (VR)

Virtual reality's fundamental properties can be utilized to aid in the educational process. Virtual reality technology's high level of communication: many people learn via practice. Clients in immersive virtual reality settings are engaged inside the virtual world thanks to specific input/output equipment. It is a helpful feature for various applications, such as architectural instruction, where a feeling of scale is critical for understanding the influence of a building's design on the external environment and its occupants. Virtual reality systems have inherent flexibility due to the software that supports the virtual world. Depending on the software programmed, a virtual reality device may be utilized in various ways. As a result, it may be used in multiple educational settings.

### 3.4. Prediction of Student Performance

#### 3.4.1. Fuzzy-Based Tweakable CNN-LSTM-AM

Fuzzy-based tweakable CNN is utilized in feature film production because it focuses on the most visible visual characteristics. LSTM, which has the property of rising with time, is commonly used in time-series analysis. An essential feature of AM is that it incorporates time-series data's previous elements into the output findings. It would be more customary to use it after LSTM to improve prediction performance.

*(1) The Fuzzy-Based Tweakable CNN-LSTM-AM Training Procedure*. The fuzzy-based tweakable CNN-LSTM-AM training process is shown in Figure 3.

  Step 1. The information required for fuzzy-based tweakable CNN-LSTM-AM education has been input.
  Step 2. Because there is significant variance across the data, *Z*-score normalization is utilized to equalize it. This makes it easier to train the model.
  Step 3. At this stage, the weights and biases of all layers of the fuzzy-based tweakable CNN-LSTM-AM are set to zero.
  Step 4. Convolution and pooling layers are used to send the incoming data to the CNN layer, which extracts the characteristics of the input data and calculates the return value.
  Step 5. The CNN layer's result is then determined using the LSTM layer's hidden layer, and the final solution is computed.
  Step 6. Running the final output of the LSTM layer via an AM layer calculation yields a value.
  Step 7. We must first calculate the AM layer's result before getting to the model's output.
  Step 8. The output layer's resulting value is compared with the actual data collection price, and the relevant error is calculated.
  Step 9. Determine whether the forecasting process' aim has been met: a positive conclusion is stated once a certain number of iterations have been completed, the weight has fallen below a certain threshold, and the prediction error rate has decreased below a certain point. When at least one of the requirements for completion has been met, the training will be completed. If this is not the case, training will continue as usual.
  Step 10. It returns to step 4 to continue training the infrastructure, but this time in the other direction, spreading the mistake backwards.
 
Figure 4 depicts the fuzzy-based tweakable CNN-LSTM-AM prediction procedure.
  Step 1. The essential data are input to produce a forecast.
  Step 2. All of the data in the input have been normalized.
  Step 3. Based on the normalized data, the trained fuzzy-based tweakable CNN-LSTM-AM predicts the target value.
  Step 4. The fuzzy-based tweakable CNN-LSTM-AM creates the normalized output to restore data scalability. The normalized value's actual data are returned.
  Step 5. To complete the prediction method, the regenerated results are delivered.

RETRACTED

### 3.5. Optimization

#### 3.5.1. Grey Wolf Optimizer

GWO is a newly developed SI algorithm that has demonstrated solid and sophisticated search abilities by following the leadership of three top swarming leaders. Its architecture is to make the transition from investigation to exploitation as easy as possible. Despite these benefits, the initial GWO algorithm still is vulnerable to optimal global trapping due to its searching bias, particularly towards the source of the coordinate system and searching diversity limits. Furthermore, during the duration of the research, the fixed and uniform distribution of authority among the top three wolves opposes the wolf society's hierarchy division method in principle, limiting the potential to fine-tune around the discovered global optimum answer. This study suggests four unique ways to remove the constraints above and improve the initial GWO computation global search and localized application. To begin, a stochastic modification of the research speed *a*^2^ is proposed to replace *a* and speed up the shift from research to harvest. During the investigation, the goal is to keep the search region from shrinking while focusing on the potential area surrounding the wolf leader during the exploit. Second, fluid yet constrained weights are produced using a chaotic sine system. The goal is to mimic benign contests for wolf pack leadership among some of the three dominant wolves *α*, *β*, and*δ*. As a result, a balance may be struck between promoting good person's management while spreading the diversions of the 2nd and 3rd best solutions. Also presented is a decelerated odd functional with diminishing magnitude. To speed up the high converge process, the next stage is to install a fine-tuning local search mechanism around the swarm leadership. Finally, the Cauchy fly is employed to improve the top three wolves' health and kill beyond early stasis in each iteration.  Algorithm 1 provides an essential pseudo-code for the suggested GWO version.

RETRACTED

## 4. Result

This study uses a fuzzy-based tweakable convolution neural network (FT-CNN-LSTM-AM) technique to investigate the significance of AI in mathematical education. This project employs artificial intelligence in the classroom setting of mathematics instruction and uses student data. It is tested to see whether it can accurately forecast how well students will do in their mathematics classes.

### 4.1. Learning Rate

The learning rate is a parameter that specifies the step length in an optimization process at every repetition as it moves forward towards an error function optimum.  Figure 5 compares the pace of learning for the current work and the new project.

When compared to previous research (“logistic regression analysis (LRA), artificial neural network (ANN), fully connected network (FCN), the adaptive neuro-fuzzy inference system (ANFIS), and conditional random field (CRF)”), the proposed method has the more excellent learning rates.

### 4.2. Student Achievement

The number of learning resources a pupil can learn in a particular period is known as student achievement. Every education level does have its own set of goals and criteria, which teachers are responsible for conveying to the pupils.  Figure 6 depicts a comparison of student achievement for existing and proposed work.

Prior studies (“logistic regression analysis (LRA), artificial neural networks (ANNs), fully connected network (FCN), adaptive neuro-fuzzy inference system (ANFIS), and conditional random fields (CRFs)”) found that the suggested technique had a better student achievement when compared to these methods. The students have a teaching method, instruction for education, house, parental participation, and a belief that all learners can understand whether we use the recommended approach.

### 4.3. Percentage of Respondents

The number of respondents could be computed by dividing the number of completed responses and replies by the total number of people that saw or began the study. To get a %, the final number is multiplied by 100 and divided by 100. A response rate of at most 50% is considered excellent. The percentage of responders for current and prospective work is shown in Figure 7.

RETRACTED

### 4.4. Math Task Accuracy

The measurement of accuracy and error-free: a number described as having a relative accuracy of because its true value might be between 99 and 101, as opposed to a number represented as having a relative accuracy (so, its actual value might be anything from 98 to 102 points).  Figure 8 compares math task accuracy for existing and proposed work.

### 4.5. Problem-Solving Skill

Problem-solving abilities assist you in figuring out why something is occurring and how to fix it. It is among the essential skills that businesses look for in job candidates. Defining the problem, troubleshooting, executing these alternatives, and assessing their efficacy are stepped in the problem-solving process.  Figure 9 depicts the problem-solving skill of the proposed work.

When compared to previous research (“logistic regression analysis (LRA), artificial neural network (ANN), fully connected network (FCN), adaptive neuro-fuzzy inference system (ANFIS), and conditional random field (CRF)”), the suggested strategy has a higher degree of problem-solving skill. Artificial intelligence can help primary school students improve their math skills. It enhances the capacity to handle situations analytically and rationally and is aided by problem-solving in math. It enhances the capacity to handle situations analytically and rationally and is aided by problem-solving in math, the knowledge to plan and arrange things, and data processing abilities.

## 5. Discussion

In LRA Bahadir [21], a common belief is that the relationship between the dependent and independent variables is always spine-like. Moreover, it measures how well a prediction (coefficient size) performs, as well as its directional connection (positive or negative). If the quantity of observations is lower than the number of variables, logistic regression must not be utilized; otherwise, overfitting might happen. ANN Al-Ghamdi et al. [22] is plagued with undefined DRG payment system behavior. There is no explanation for why or how ANN produces a probing resolution. This harms the level of confidence users have in the network. Thus, ANFIS's Stojanovic et al. [23] “black box” drawbacks—the incapacity to justify decisions (lack of transparency) and the difficulty of learning in fuzzy logic—have indeed been overcome consequently. In CRF Liu et al. [24] algorithm's learning phase's computing cost is by far CRF's biggest drawback. To train a model once more when fresh learning evidence is accessible is much more challenging for this feature. In FCN Hooda et al. [25], a 1×1 convolution operation replaces the final convolutional layer inside the FCN topology, and a last picture with the exact dimensions as the input feature map is created. So, we propose VR technology that encourages kids to study and grow in their lives and enhances the educational value—aids in comprehending complex ideas, disciplines, or theories. There will be no interruptions during studying. Pupils' inventiveness is boosted. The effectiveness with which students acquire information is improved.

RETRACTED

## 6. Conclusion

In this study, we have widely focused on the role of AI in mathematics development and the education of intelligent tutoring systems for Internet educational experiences. We concluded that with the implementation of Internet education, students' learning capacities improved tremendously. Most elementary school pupils are enticed to acquire fundamental mathematical notions more actively by natural math challenges in the form of enhanced gaming tactics. Educators are also utilizing these systems in the syllabus, which can benefit all other educators who are not now using processes. Numerous visualizations improve information retention and transmission of core ideas throughout time. In elementary school, comparing various techniques or tactics kids use to resolve an issue increases natural competition and advanced mathematical thinking. These intelligent machines motivate students to devise new computational solutions to tackle the problem successfully. It encourages pupils to develop multifunctional abilities that lead to deeper learning. These technologies promote Internet learning as opposed to the conventional college course learning. Speech sound recognition techniques and natural language are used by teaching bots to help students understand the value of augmented worlds in education. Reconnection and presentation of detailed information are used to benefit from such platforms. Through participatory exploration, physics, chemistry, and statistics are made more intelligible for students. Establishing automation laboratories in academic institutions is a novel technique of teaching actual computers rather than virtual devices that can mimic all human abilities. AI has become the necessity of the moment to future generations as it attempts to transcend human observation or intellect more precisely.

## Figures and Tables

**Figure 1:** Mathematical education using artificial intelligence.

RETRACTED

**Figure 2:** Proposed methodology.

**Figure 3:** Fuzzy-based tweakable CNN-LSTM-AM training procedure.

**Figure 4:** Fuzzy-based tweakable CNN-LSTM-AM prediction procedure.

**Figure 5:** Comparison of the learning rate for existing and proposed work.

**Figure 6:** Comparison of student achievement for existing and proposed work.

**Figure 7:** Comparison of percentage of respondents for existing and proposed work. When compared to previous research (“logistic regression analysis (LRA), artificial neural network (ANN), fully connected network (FCN), adaptive neuro-fuzzy inference system (ANFIS), and conditional random field (CRF)”), the proposed method has the more significant percentage of respondents.

**Figure 8:** Comparison of math task accuracy for existing and proposed work. When compared to previous research (“logistic regression analysis (LRA), artificial neural network (ANN), fully connected network (FCN), adaptive neuro-fuzzy inference system (ANFIS), and conditional random field (CRF)”), the suggested strategy has a higher degree of math task accuracy.

**Figure 9:** Problem-solving skill.

**Algorithm 1:** The GWO model

**Table 1:** Dataset description.

	Variable	Mean	Std. dev.	Min	Max
Full sample (*n* = 23,143)					
1.	Gender (1 = male)	0.55	0.40	0	1.10
2.	Age (years)	12.35	1.22	8.00	15.00

Guizhou and Jiangxi sample (*n* = 16,253)					
3.	At school, students live (1 = yes)	0.15	0.33	0	1.01
4.	Socioeconomic disadvantage (1 = yes)	0.45	0.55	0	1.01

Shaanxi sample (*n* = 5,700)					
5.	Gender (1 = male)	0.57	0.57	0	1.10
6.	Age (years)	10.88	1.23	8.00	15.20
7.	Type of hukou (1 = rural hukou)	0.87	0.37	0	1.00

Guizhou sample (*n* = 2,658)					
8.	Gender (1 = male)	0.55	0.52	0	1.10
9.	Age (years)	11.48	1.50	7.00	15.00
10.	At school, students live (1 = yes)	0.08	0.24	0	1.10
11.	Socioeconomic disadvantage (1 = yes)	0.54	0.51	0	1.10

Jiangxi sample (*n* = 13,995)					
12.	Gender (1 = male)	0.56	0.52	0	1
13.	Age (years)	11.46	1.09	7.00	15.00
14.	At school, students live (1 = yes)	0.20	0.36	0	1
15.	Socioeconomic disadvantage (1 = yes)	0.52	0.52	0	1

## Data Availability

The data used to support the findings of this study are available from the corresponding author upon request.
